RETRACTED

# Identifying the Effect of Nuanxin Capsules on Myocardial Injury Induced by Chronic Hypoxia via Network Pharmacology Analysis and Experimental Validation

**DOI:** 10.1155/2022/2399462

**Published:** 2022-10-04

**Authors:** Zhexing Mai, Ye Fan, Jin Ma, Tiantian Lou, Shiyu Ma, Xu Zou

**Affiliations:** ^1^The Second Affiliated Hospital of Guangzhou University of Chinese Medicine, Guangzhou 510120, China; ^2^The Second Clinical College of Guangzhou University of Chinese Medicine, Guangzhou 510120, China; ^3^Guangdong Provincial Hospital of Chinese Medicine, Guangzhou 510120, China; ^4^State Key Laboratory of Emergency of Chinese Medicine, Guangdong Provincial Hospital of Chinese Medicine, Guangzhou 510120, China; ^5^Intensive Care Unit of Dongguan Hospital, Guangzhou University of Chinese Medicine, Guangdong 523000, China

## Abstract

Nuanxin capsule (NX), an in-hospital preparation of Guangdong Provincial Hospital of Chinese Medicine, has been used in heart failure (HF) treatment for 15 years, but its mechanism and protective effect have not been investigated. This study was aimed at exploring the mechanism and protective effect of NX on HF treatment via network pharmacology analysis and experimental validation. Network pharmacology analysis predicted that NX was involved in the regulation of response to apoptotic process and hypoxia via protecting cellular damage and mitochondrial dysfunction against chronic hypoxia. Its mechanism may be involved in the regulation of the PI3K-Akt signaling pathway, HIF-1 signaling pathway, AMPK signaling pathway, and MAPK signaling pathway. Experimental validation indicated that NX was capable of improving cellular viability, restoring cellular morphology, and suppressing cellular apoptosis cellular. NX also exerted cardioprotection by inhibiting mitochondrial membrane potential injury and protecting mitochondrial respiratory and energy metabolism in a chronic hypoxia cellular model, which was consistent with the results of network pharmacology prediction. In addition, the screened active compounds of NX did have a good binding with their key targets, indicating NX may exert protective effect through multicompounds and multitargets. In conclusion, NX had a protective effect on HF through cellular and mitochondrial protection against chronic hypoxia via multicompounds, multitargets, and multipathways, and its mechanism may be involved in modulating the PI3K-Akt signaling pathway, HIF-1 signaling pathway, AMPK signaling pathway, and MAPK signaling pathway.

## 1. Introduction

Heart failure (HF) has become a major public health problem, threatening human health globally. It affects approximately 23 million people and is accompanied by increasing mortality and hospitalization rates [1]. Chronic and intermittent hypoxia is mainly responsible for the development of pulmonary hypertension [2], which induces right ventricular hypertrophy in the long term [3], leading to a vicious cycle in the impairment of right ventricular performance and failure, eventually leading to death [4, 5]. Mechanistic studies have revealed that HF is associated with oxidative stress, inflammation, mitochondrial dysfunction, and calcium overload, *inter alia*, due to chronic hypoxia [6]. Despite advances in drug development, effective therapies for improving HF prognosis by targeting chronic hypoxia are still lacking [7].

RETRACTED

Traditional Chinese medicine contains multicompounds and exerts therapeutic effects on HF by targeting multiple targets through multiple pathways; it has been proven to be effective and safe in preventing and treating cardiovascular diseases in China [8]. The Nuanxin capsule (NX), an in-hospital preparation of Guangdong Provincial Hospital of Chinese Medicine prescribed by Professor Tietao Deng, has been used in clinical practice for 15 years and has a stable and safe effect in chronic HF [9]. The NX consists of *Red Ginseng*, *Radix Aconiti Lateralis Preparata*, *Poria*, and *Coix seed*, which exert effects of warming heart qi by alleviating water retention, expelling blood stasis in the heart vessels, strengthening the spleen, and nourishing the heart in terms of Chinese medicine [10]. Clinical research has revealed that NX effectively regulates the NYHA functional class, plasma BNP, and 6 min walking distance to relieve the symptoms of chronic HF and improves exercise tolerance and quality of life [11]. A systematic review has shown that NX, combined with conventional drug therapy, significantly decreases mortality and readmission rates [12]. Our previous study revealed that NX could inhibit the myocardial injury caused by oxidative stress through the AMPK pathway [13], but the verification of whether NX has a pharmacological effect on myocardial injury induced by chronic hypoxia in HF is still absent.

As NX has been identified as a multiple compound using ultraperformance liquid chromatography quadrupole time-of-flight tandem mass spectrometry (UPLC-Q-TOF-MS) method in our previous study, thus in this study, we further predicted the pharmacological effect and mechanism of the NX on HF based on the identified multicompounds using network pharmacology and molecule docking analyses. Then, the pharmacological effect of NX *in vitro* was further validated using a chronic hypoxia cellular model.

## 2. Materials and Methods

### 2.1. Drugs and Reagents

Rat cardiomyocyte H9c2 cells were purchased from Cell Bioscience Inc. (Shanghai, China). Nuanxin capsule is composed of *Red Ginseng*, *Radix Aconiti Lateralis Preparata*, *Poria*, *and Coix seed* and was purchased from Guangdong Provincial Hospital of Chinese Medicine (production batch number: 190501, each capsule weighs 0.5 g). Dulbecco's Modified Eagle Medium (DMEM, USA), fetal bovine serum (FBS, Australia), 0.25% Trypsin-EDTA Solution, 3-(4,5-dimethylthiazol-2-yl)-2,5-diphenyltetrazolium bromide (MTT, Cat. No. #M5655), and phosphate-buffered saline (PBS, USA) were purchased from Gibco (Grand Island, NY, United States), and Annexin V-FITC Apoptosis Detection Kit (No. C1062L) and mitochondrial membrane potential assay kit with JC-1 (JC-1, No. C2006) were purchased from Beyotime Biotechnology Co., Ltd. (Shanghai, China). Seahorse XF Cell Mitochondrial Stress Test Kit (103010-100) was purchased from Agilent (United States).

RETRACTED

### 2.2. Collection of Compounds Contained in NX

The compounds were identified by the UPLC-Q-TOF-MS method in our previous study [13]; thus, a total of 23 compounds of NX were collected from our previous research, their names were standardized by the PubChem database (https://pubchem.ncbi.nlm.nih.gov/), and the 2D structures of these compounds were downloaded from the PubChem database.

### 2.3. Collection of Targets of Identified Compounds

The targets of compounds contained in NX were collected from Traditional Chinese Medicine Systems Pharmacology Database and Analysis Platform (TCMSP, https://old.tcmsp-e.com/tcmsp.php) and SwissTargetPrediction Platform (http://www.swisstargetprediction.ch/).

### 2.4. Collection of Heart Failure Targets

The key words “Heart failure”, “Cardiac Failure”, and “Heart Decompensation” were used to retrieve the targets related to HF in the OMIM database (https://www.omim.org/) and the GeneCards database (http://www.genecards.org/) with a relevance score no less than 5.

### 2.5. Intersection Target Screened by Venn Analysis

The intersection targets between identified compounds of NX and HF disease targets were screened by Venn analysis, which were seen as targets of NX-identified compounds that had a potential pharmacological effect on HF.

### 2.6. PPI Network Construction and Core Target Selection

The UniProt IDs of candidate targets were matched from the UniProt database (https://www.uniprot.org/) and uploaded to the STRING database (https://cn.string-db.org/) to acquire protein-protein interaction (PPI) network, with a score no less than 0.75. Cytoscape_3.9.1 software was utilized to visualize the PPI network. Top 20 targets with the highest degree value were regarded as core targets.

### 2.7. Gene Ontology Annotation (GO) and Kyoto Encyclopedia of Genes and Genomes (KEGG) Pathway Enrichment Analysis

The GO enrichment analysis on the intersection targets was conducted through the DAVID platform (https://david.ncifcrf.gov/), including cellular component (CC), biological process (BP), and molecular function (MF). KEGG pathway enrichment analysis on the intersection targets was also performed through DAVID platform. The item with *p* value < 0.05 was selected, and the top 20 items of GO enrichment and the top 40 items of KEGG pathway enrichment were visualized by enrichment bar or bubble plots.

RETRACTED

### 2.8. Component–Disease–Target-Potential Pathway Network Construction

The intersection targets, identified compounds, diseases, and pathways were introduced into Cytoscape 3.9.1 software to visualize the possible mechanism of NX against HF, revealing the distribution characteristics among intersection targets, identified compounds, diseases, and pathways. Key targets and key pathways were selected according to the connection degree.

### 2.9. Molecular Docking Analysis on Screened Targets and Identified Compounds of NX

Five key targets enriched in the potential pathways were selected, their structures were downloaded from the PDB database (https://www.rcsb.org/), and the PyMOL software was used to embellish the protein structures via affixing hydrogen atoms and removing water molecules. Finally, the modificatory protein structures and 3D structures of the homologous small molecules were downloaded from the PubChem database (https://pubchem.ncbi.nlm.nih.gov/) and were submitted to Schrödinger software to perform molecular docking. A binding energy explained that the ligand could spontaneously bind with the receptor, and the lower binding score indicated the stronger binding ability.

### 2.10. Cell Culture and Treatment

Rat cardiomyocyte H9c2 cells were cultured in DMEM supplemented with 10% FBS. The culture medium was replaced once every 2-3 days, and the cells were passaged at a ratio of 1 : 3. The cardiomyocytes were assigned into 5 groups: (a) control group, (b) chronic hypoxia group, (c) chronic hypoxia group+low-dose NX (NX-L) group, (d) chronic hypoxia group+median-dose NX (NX-M) group, and (e) chronic hypoxia group+high-dose NX (NX-H) group. The method of hypoxia model was as follows: when the cell confluency density reached about 80% in a 37°C, 5% CO_2_ incubator, the original medium was discarded, then rinsing the cells with PBS and replacing the original medium with no glucose and serum-free medium for each group except the control group. NX groups were treated with different doses (2, 4, and 6 mg/mL) at the time when modeling began; finally, the cells in the chronic hypoxia group and NX groups were transferred to a 37°C, 0.1% O_2_, 5% CO_2_, and 95% N_2_ for 24 h hypoxia.

RETRACTED

### 2.11. Cytotoxicity of NX on Cells

Cytotoxicity of NX and cellular proliferation were detected by MTT assay. Cells were cultured in 96-well plates at a density of 6000 per well. When the cell confluency was 80%, the original medium was removed and the cells were washed twice with 1x PBS. After treatment and modeling, MTT solution (0.5 mg/mL) was added to each well after removing the drug solution, and cells were incubated in a 37°C incubator for 4 hours. Finally, the MTT solution was removed, 100 *μ*L of DMSO solution was added to each well for 10 min at room temperature to dissolve the formazan crystals. The OD value of each well indicating cellular viability was recorded at 570 nm using a microplate reader (Thermo Fisher Scientific, Multiskan FC, USA); the cytotoxicity of NX on cells was represented by cellular viability.

### 2.12. Cellular Impaired Morphology Observation

In cellular morphology observation, after cell culture and treatment, cellular morphology was imaged by a fully automatic inverted fluorescence microscopic analysis system (ECLIPSE Ti2-E, Nikon, Japan).

### 2.13. Cellular Apoptosis Assay

The cell apoptosis rate of H9c2 cells was measured by Annexin V-FITC Apoptosis Detection Kit according to the manufacturer's instructions. After receiving different treatments, the culture medium was aspirated and cells were collected; then, cells were stained with 195 *μ*L Annexin V-FITC binding solution (1x) and 10 *μ*L Annexin V-FITC plus 5 *μ*L propidium iodide (PI) solution for 15 min at room temperature. Finally, the cell apoptosis rate was immediately analyzed by flow cytometry (Agilent, NovoCyte Quanteon, USA).

### 2.14. Mitochondrial Membrane Potential (*ΔΨ*m) Assay

The effects of different concentrations of NX working solution on the mitochondrial membrane potential of H9c2 cells were evaluated by flow cytometry using the mitochondrial membrane potential assay kit with JC-1 (Beyotime Biotechnology Co., Ltd., China). The preprocessing method was performed according to the manufacturer's protocol. After treatment, 500 *μ*L JC-1 staining solution was added to each group of cell samples for 20 min incubation at 37°C, and then, it was washed twice with JC-1 buffer solution. Finally, the injury degree of *ΔΨ*m was immediately detected by flow cytometry (Agilent, NovoCyte Quanteon, USA).

### 2.15. Mitochondrial Respiration by Oxygen Consumption Rate (OCR) Assay

Mitochondrial respiration by oxygen consumption rate (OCR) in each group was measured by Seahorse XFe Cell Mitochondrial Stress Test Kit. Cells were plated overnight in 24-well plates at a density of 4 × 10^4^; then, the cells were cultured and treated. After treatment, the medium was replaced with XFe assay medium dissolved with 10 mM glucose, 1 mM pyruvate, and 2 mM glutamine. Then, the cell plate was placed in a CO_2_-free incubator at 37°C for 1 h, and the stock solutions of oligomycin (complex V inhibitor), FCCP (respiratory uncoupler), and rotenone/antimycin A (inhibitor of complex I and complex III) were added to the A, B, and C ports, respectively. Basal respiratory, spare respiratory capacity, mitochondrial maximal respiration, and adenosine triphosphate (ATP) production of cells were measured through a Seahorse XFe24 analyzer (Agilent Seahorse, USA). Finally, the OCR value was normalized by CCK8 detection.

RETRACTED

### 2.16. Statistical Analysis

The experimental data were expressed as the mean ± SEM, and one-way ANOVA for comparing the difference among groups was performed using GraphPad Prism Software (version 7, GraphPad Prism Software, San Diego, CA, USA). Postmultiple comparison was conducted by the Bonferroni test. The experimental data were repeated from 3 independent experiments; *p* < 0.05 indicates significant statistical difference.

## 3. Results

### 3.1. Identified Compounds of NX

A total of 23 compounds were identified by the UPLC-Q-TOF-MS method. Apart from two compounds (Meringenin and 20(S)-NG-R2), which had no record about their information in the PubChem database, 21 compounds were collected for latter analysis (see Table 1).

### 3.2. Intersection Targets of Identified Compounds of NX Related to HF

401 protein targets of identified compounds of NX were harvested via SwissTargetPrediction website platform, and 120 targets were collected from the TCMSP database. After duplication, a total of 481 targets were selected. In addition, 12017 and 1279 HF targets were obtained from the GeneCards database and OMIM database, respectively, and 12063 HF targets were screened after duplication. Finally, Venn analysis screened 454 intersection targets of identified compounds of NX related to HF (see Figure 1(a)).

### 3.3. PPI Network of NX-HF Intersection Targets and Filtrating Core Targets

The PPI data containing 7883 interactions were downloaded from the STRING database; 3963 interactions containing 454 targets were selected with a combined score no less than the median (0.601). The PPI network consists of 438 nodes and 3963 interaction edges (Figure 1(b)). 20 targets with the largest degree value were considered the core targets, which were calculated by the built-in tool of Cytoscape_3.9.1 software, including *Tumor suppressor p53/oncoprotein Mdm2*, *Serine/threonine protein kinase AKT*, and *Axin1/beta-catenin* (see Table 2).

RETRACTED

### 3.4. Results of Gene Ontology (GO) Annotation Enrichment

GO functional annotation and KEGG pathway analysis were performed on 454 targets in the PPI network. In the cellular components (CC), targets were closely enriched on the cellular membrane, cell surface, and mitochondrion (see Figure 2(a)). Targets enriched in the biologic process (BP) included response to apoptotic process, response to hypoxia, and cellular response to hypoxia (see Figure 2(b)). At the molecular function (MF) level, the targets were mainly related to protein binding, ATP binding, and protein kinase activity (see Figure 2(c)). The GO enrichment analysis revealed that most of the candidate targets of NX were associated with cellular membrane and mitochondria in response to hypoxia and ATP binding, suggesting that NX may exert its effect through mitochondria and cellular function against chronic hypoxia in HF. Thus, our validated experiment was focused on the cellular and mitochondrial function through a chronic hypoxia-induced cellular model to verify the pharmacological effect of NX.

### 3.5. Results of Kyoto Encyclopedia of Genes and Genomes (KEGG) Pathway Enrichment

KEGG pathway analysis showed that the top pathways with higher degree included the PI3K-Akt signaling pathway, HIF-1 signaling pathway, AMPK signaling pathway, MAPK signaling pathway, and apoptosis signaling pathway (see Figure 3(a)). When we conducted the KEGG enrichment analysis on the top 20 core targets, the enrichment results still included the PI3K-Akt signaling pathway, HIF-1 signaling pathway, AMPK signaling pathway, MAPK signaling pathway, and apoptosis signaling pathway (see Figure 3(b)). Thus, the PI3K-Akt signaling pathway, HIF-1 signaling pathway, AMPK signaling pathway, MAPK signaling pathway, and apoptosis signaling pathway were considered the potential pathways of NX against HF (see Figures 3(c) and 3(d)).

### 3.6. NX Improved Cellular Injury Induced by Chronic Hypoxia

MTT assay suggested that NX had no cytotoxicity on H9c2 cells as there was no statistical difference among the groups (NX0.25, NX0.5, NX1, NX2, NX4, NX6, and NX8 mg/mL) compared with control group (see Figure 4(c)). In addition, as shown in Figure 4(b), the cell viability in the chronic hypoxia group was significantly reduced, but cellular viability increased as the NX concentration increased, while when the concentration was up to 6 mg/mL, it showed a decreased trend compared with 4 md/mL; thus, 1, 2, and 4 mg/mL were selected for later experiments for they had the best effect on improving the cellular viability. As shown in Figure 4(a), the cells in the chronic hypoxia group were impaired, represented by sparse arrangement, and cell necrosis was indicated as white, bright aperture and round shaped compared with the control group. However, in the 1, 2, and 4 mg/mL NX groups, the cellular morphology was restored with regular and tight arrangement, and white bright aperture was decreased. All the above suggested that NX could restore the cellular morphology damage and alleviate cellular injury induced by chronic hypoxia.

RETRACTED

### 3.7. NX Alleviated Cellular Apoptosis Induced by Chronic Hypoxia

Figure 5(a) showed the results of early apoptosis, late apoptosis, and normal cells in each group. As shown in Figure 5(b), the ratios of normal cells in the chronic hypoxia group were significantly decreased compared with those in the control group, but with NX treatment, the ratio in the 1, 2, and 4 mg/mL groups gradually increased by comparing with that in the chronic hypoxia group. Figures 5(c) and 5(d) reveal that the early apoptosis rate and late apoptosis rate in the chronic hypoxia group were significantly increased compared with those in the control group, but in the NX group, they were decreased with statistical difference; the results indicated that NX could inhibit the apoptosis in H9c2 cells induced by chronic hypoxia.

### 3.8. NX Inhibited Mitochondrial Membrane Potential (*ΔΨ*m) Injury Induced by Chronic Hypoxia

To determine whether NX protected mitochondria damage in response to chronic hypoxia, mitochondrial membrane potential (*ΔΨ*m) was detected by JC-1 staining.  Figure 6(a) shows the red fluorescence weakened and the green fluorescence strengthened because of the damage of cells in the chronic hypoxia group compared with the control group, but with the treatment of NX, the red fluorescence strengthened and the green fluorescence weakened, indicating the function of mitochondria was restored by NX. The result was further confirmed by mitochondrial membrane potential flow cytometer detection; as shown Figures 6(b) and 6(c), the rate of cells with decreased *ΔΨ*m in the chronic hypoxia group significantly increased compared with that in the control group, while in the 1, 2, and 4 mg/mL groups, it was decreased with statistical difference. All the above revealed that NX could inhibit mitochondrial membrane potential (*ΔΨ*m) injury induced by chronic hypoxia.

### 3.9. NX Protected Mitochondrial Respiratory from Chronic Hypoxia-Induced Injury

To evaluate the protective effects of NX on mitochondrial respiratory, the oxygen consumption rate of H9c2 cells was examined (see Figure 7).  Figure 7(a) shows that the OCR valve changed at different time points.  Figure 7(e) shows that the basal respiration in the chronic hypoxia group decreased, but it increased after NX treatment. Figures 7(b)–7(d) show the same trend that, compared with the control group, chronic hypoxia decreased the ability of maximal respiratory, spare respiratory capacity, and ATP production, but it was gradually restored in the NX, indicating that NX protected mitochondrial respiratory from chronic hypoxia-induced injury.

RETRACTED

### 3.10. Molecular Docking Analysis

We conducted molecular docking analysis between the screened active compounds and predicted key targets, providing evidence support for network pharmacology prediction. The results showed that Apigenin had a strong binding ability with HIF1A (docking score = −5.96), AKT1 (docking score = −5.765), GSK3B (docking score = −6.327), and SLC2A4 (docking score = −7.912). Naringenin had a strong binding ability with MAPK3 (docking score = −6.749) and GSK3B (docking score = −6.749). Acacetin had a strong binding ability with GSK3B (docking score = −6.788), Aurapten had a strong binding ability with GSK3B (docking score = −6.991), and Oxypeucedanin had a strong binding ability with GSK3B (docking score = −6.06) (see Table 3). The docking results suggested that the bioactive components of NX had good binding with key targets, which indicated a strong reliability of our prediction. The docking structures are displayed in Figure 8.

## 4. Discussion

Heart failure is one of the most common clinical diseases, accounting for abundant morbidity and mortality worldwide. At present, even though there is large progress in drug management, it is insufficient to halt HF progression [14, 15]; thus, additional therapeutic approaches that focus on improving the prognosis of HF should be developed. NX is a commonly used, patented prescription and clinical Chinese medicine against HF with a satisfactory curative effect [16]. However, the effects and underlying mechanisms of NX on HF remain unknown. This study integrated chemical constituents, network pharmacology, and *in vitro* pharmacodynamic experiments to investigate the cardioprotective effects of NX on HF.

NX contains 4 kinds of herbs with multicompounds; a variety of chemical reactions can occur during the extraction and purification process. Therefore, in order to clarify the chemical composition of NX, we collected a composition identified by the UPLC-Q-TOF-MS method to predict the therapeutic mechanisms of NX on HF. 21 active components were obtained, including naringenin, and ginsenoside rb2. Naringenin, a flavonoid, has been demonstrated to exert cardioprotective effects [17]. Yu et al. [18] proved naringenin could improve the mitochondrial function of cardiomyocyte damaged by ischemia-reperfusion in *vitro* via inhibiting oxidative stress damage and enhancing mitochondrial biogenesis. Moreover, the cardiac function of Sprague-Dawley rats undergoing MI/R surgery improved after treatment with naringenin. Ginsenoside rb2 also has the potential to protect against HF. Wang et al. [19] found that ginsenoside rb2 was the activator of sirtuin type 1 (SIRT1) and it could enhance the deacetylation activity of SIRT1, increase ATP content, inhibit the formation of intracellular reactive oxygen species, and regulate the activity of manganese superoxide dismutase to protect H9c2 cardiomyocytes from oxidative damage. Several single chemical compounds have been proven to have pharmacological protection in *vivo* or *vitro*, but it still lacks verification on the pharmacological effect of NX as a mixture of multicompounds against HF.

RETRACTED

Network pharmacology analysis indicated that the NX was involved in the response to apoptotic process, response to hypoxia, and the mitochondrial response to hypoxia and was involved in cellular components including the cellular membrane, cell surface, and mitochondria. These indicate that NX may exert its antihypoxia effect and protection through inhibiting cellular injury and mitochondrial dysfunction. Hypoxia is a common feature in the pathophysiology of various cardiovascular diseases [20]; it can disturb vascular homeostasis and result in smooth muscle cell hyperplasia and mitochondrial dysfunction in the vessel graft [21]. Hypoxia can induce cardiomyocyte injury and apoptosis, which contribute significantly to cardiac dysfunction [22]. Acute cardiac dysfunction leads to altered cardiomyocyte mechanics, perturbations in mitochondrial sarcomere architecture, and deficits in mitochondrial function, which can lead to the activation of apoptosis and HF [23]. Cardiac hypertrophy and apoptosis are major characteristics of early-stage HF, and the activation of apoptotic pathways contributes to cardiomyocyte loss and subsequent cardiac dysfunction [24]. Impeding cardiomyocyte apoptosis plays a novel role in modulating cardiomyocyte protection [24]. Additionally, the inhibition of cellular apoptosis can delay or prevent the development of HF [25–27]. In the present study, we found that NX could restore cellular morphology and alleviate cellular injury induced by chronic hypoxia. It was further verified that the NX substantially decreased the early and late apoptosis rates induced by chronic hypoxia, suggesting that NX protected cardiomyocytes from apoptosis.

Mitochondrial dysfunction has been implicated in the development of HF due to myocardial hypoxia [28]. The inability of oxidative metabolism to generate and transfer energy is considered the primary mechanism linking to mitochondrial dysfunction and contractile failure [29]. Mitochondria affects cardiomyocyte physiology by regulating ATP synthesis and oxygen consumption. The maintenance of cardiac mitochondrial function and integrity is critical in the treatment of HF [30]. Numerous clinical trials of agents have sought to improve mitochondrial function by acting on different aspects of mitochondrial function [31–33]. Therapeutic agents that improve mitochondrial function are likely to enhance both cardiac function and peripheral oxygen utilization [34]. The mitochondria are important for aerobic respiration and energy exchange. As a highly energy-consuming organ, the heart needs to consume a large amount of ATP daily to ensure a normal energy supply. Cardiac injury is accompanied by insufficient ATP synthesis, decreased mitochondrial membrane potential, and weakened mitochondrial respiratory function. Modulation of mitochondrial function is a new approach for cardiovascular disease treatment [34, 35]. In the present study, we found that NX restored mitochondrial function by improving the mitochondrial membrane. It was further verified that NX substantially increased maximal respiratory capacity, spare respiratory capacity, and ATP production, suggesting that NX promoted energy supply to the cardiomyocytes, which was consistent with predicted results of the network pharmacology analysis.

RETRACTED

The PPI network analysis predicted that TP53 might play an important role in NX against HF. TP53 is upregulated in the failing myocardium of humans [36]. High concentrations of TP53 induce an increase in glycolysis, possibly by increasing the expression of TP53-induced glycolysis and apoptosis regulators (TIGAR). In addition, knockout of TIGAR improves energy metabolism and protects heart function from HF-associated damage [37]. Activated Akt inhibits apoptosis of cardiomyocytes and improves their survival under hypoxia by enhancing the phosphorylation of the apoptosis regulator, Bcl-2 family, and GSK3B [38, 39]. However, another study suggests that persistent overexpression of activated AKT1 can lead to HF because of impaired mitochondrial oxidative capacity [40]. Cha et al. [41] concluded that the different physiological effects of AKT1 were related to the deacetylation of different pleckstrin homology domain residues. When CTNNB1 was activated in endothelial cells and cardiomyocytes, it played two different roles in cardiomyopathy. Zhu and Lu [42] reported that activated CTNNB1 in cardiomyocytes, caused by miR-423-5p inhibition, had a positive effect in alleviating cardiomyocyte apoptosis and mitochondrial dysfunction. The results of Nakagawa et al. [43] suggested that sustained activation of CTNNB1 in endothelial cells may be responsible for HF by inhibiting the signal transduction between Neuregulin and ErBb protein. In this study, it predicted that TP53, AKT1, and CTNNB1 were the core targets of NX compounds, indicating that NX may exert its pharmacological therapeutic effect against HF by targeting TP53, AKT1, and CTNNB1.

RETRACTED

The KEGG enrichment results showed that the potential targets were mostly involved in the PI3K-Akt, HIF-1, AMPK, and MAPK pathways. The PI3K-AKT pathway regulates cardiac metabolism and heart growth during pathological remodeling of HF [44, 45]. The MAPK pathway may be involved in the interaction between mitochondrial energy metabolism and systemic inflammation in injured cardiac cells [46]. It is worth noting that the PI3K-Akt and MAPK pathways are upstream of the HIF-1 pathway. Thus, we inferred that NX functions against HF mainly via the HIF-1 pathway. Similarly, the Danqi Pill reduced cardiac dysfunction and promoted cardiac glucose metabolism in postacute myocardial infarction HF rats by upregulating the expression of HIF-1*α* protein to activate the HIF-1 pathway [47]. Wang et al. [48] found that Qiliqiangxin induced cardioprotective effects, not only by upregulating HIF-1*α* and a series of glycolysis-relevant enzymes in a HIF-1*α*-dependent manner by promoting adenosine triphosphate (ATP) production, glucose uptake, and glycolysis but also by activating the downstream vascular endothelial growth factor (VEGF) pathway to increase myocardial capillary density. The role of the AMPK pathway in the therapeutic mechanism of HF has been widely studied. As an “energy regulator,” AMPK plays an essential role in regulating autophagy, cell survival, and energy metabolism [49, 50]. Previous research has indicated that empagliflozin reduces inflammatory injury by counteracting lipopolysaccharide-mediated AMPK dephosphorylation in cardiomyocytes [51]. The molecular docking analysis indicated that the ingredients of NX could bind to key HF-related targets, which suggested that NX was more likely to treat HF via these pathways.

It is worth mentioning that our study was a preliminary exploration of NX effect on HF. We collected compositional information of 21 compounds, but the quantitative determination of content required further experiments. In addition, we explored the mechanism of NX against HF via the network pharmacology and validated the cardioprotective efficacy of NX with *vitro* experiments. However, in terms of the bioactive forms of the components that may be different in *vivo* and *vitro*, our conclusions needed to be further verified with animal experiments or human trials in the future.

RETRACTED

## 5. Conclusions

In conclusion, NX had a protective effect on HF through cellular and mitochondrial protection against chronic hypoxia via multicompounds, multitargets, and multipathways; its mechanism may be involved in modulating the PI3K-Akt signaling pathway, HIF-1 signaling pathway, AMPK signaling pathway, and MAPK signaling pathway, which need to be verified in our future research.

## Figures and Tables

**Figure 1:** Intersection targets of identified compounds of NX related to HF and PPI network analysis on intersection targets. (a) Intersection targets of identified compounds of NX related to HF by Venn analysis; (b) PPI network analysis on intersection targets.

**Figure 2:** Gene ontology annotation (GO) enrichment. (a) Cellular component; (b) molecular function; (c) biological process.

**Figure 3:** Kyoto Encyclopedia of Genes and Genomes (KEGG) pathway enrichment. (a) KEGG enrichment results of core targets. (b) KEGG enrichment results of the top 20 core targets. (c) Component-disease-target-potential pathway network. (d) The target potential pathway network was enlarged in the upper figure.

**Figure 4:** Nuanxin capsule improved cellular injury induced by chronic hypoxia. (a) Cell morphology observation. (b) The effects of NX capsule on chronic hypoxia-induced H9c2 cells. (c) The cytotoxicity of NX on H9c2 cells. Data were presented as the mean ± SEM (*n* = 3). ^∗^*p* <0.05, ^∗∗^*p* < 0.01, ^∗∗∗^*p* < 0.001, and ^∗∗∗∗^*p* < 0.0001.

**Figure 5:** Nuanxin capsule alleviated cellular apoptosis induced by chronic hypoxia. (a) Cell apoptosis rate presented by flow cytometry. Q1: rate of necrotic cells/mechanical damage; Q2: late apoptosis rate; Q3: normal cell rate; Q4: early apoptosis rate. (b) Statistical analysis for normal cell rate. (c) Statistical analysis for late apoptosis rate. (d) Statistical analysis for early apoptosis rate. Data were presented as the mean ± SEM (*n* = 3). ^∗^*p* < 0.05, ^∗∗^*p* < 0.01, ^∗∗∗^*p* < 0.001, and ^∗∗∗∗^*p* < 0.0001.

**Figure 6:** NX capsule inhibited mitochondrial membrane potential (*ΔΨ*m) injury induced by chronic hypoxia. (a) Mitochondrial activity detected by JC-1 staining. (b) Mitochondrial membrane potential (*ΔΨ*m) detected by flow cytometry. (c) Statistical analysis for the rate of cells with decreased mitochondrial membrane potential (*ΔΨ*m). Data were presented as the mean ± SEM (*n* = 3). ^∗^*p* < 0.05, ^∗∗^*p* < 0.01, and ^∗∗∗^*p* < 0.001.

**Figure 7:** NX capsule protected mitochondrial respiratory from chronic hypoxia-induced injury. (a) OCR valve of mitochondrial function changed at different time points. (b) Statistical analysis for maximal respiration. (c) Statistical analysis for ATP production. (d) Statistical analysis for spare respiration capacity. (e) Statistical analysis for basal respiration. Data were presented as the mean ± SEM (*n* = 3). ^∗^*p* < 0.05, ^∗∗^*p* < 0.01, ^∗∗∗^*p* < 0.001, and ^∗∗∗∗^*p* < 0.0001.

RETRACTED

**Figure 8:** 3D docking structure and of six components docked with their predicted targets. (a) 3D docking structure of Apigenin docked with AKT1; (b) 3D docking structure of naringenin docked with AKT1; (c) 3D docking structure of Acacetin docked with GSK3B; (d) 3D docking structure of Apigenin docked with GSK3B; (e) 3D docking structure of Aurapten docked with GSK3B; (f) 3D docking structure of naringenin docked with GSK3B; (g) 3D docking structure of Oxypeucedanin docked with GSK3B; (h) 3D docking structure of Apigenin docked with HIF1A; (i) 3D docking structure of Apigenin docked with MAPK3; (j) 3D docking structure of Tuberonic acid docked with MAPK3; (k) 3D docking structure of Apigenin docked with SLC2A4.

**Table 1:** Information of identified compounds of NX by the UPLC-Q-TOF-MS method.

No.	Compound	PubChem CID	Element composition	Source
1	Apigenin-6,8-di-C-glucoside	442664	C27H30O15	Panax ginseng
2	Apigenin,7-*β*-D-glucopyranoside	5280704	C21H20O10	Panax ginseng
3	Dihydrokaempferol	122850	C15H12O6	Panax ginseng
4	Apigenin	5280443	C15H10O5	Exocarpium Citri Grandis
5	Rhoifolin	5282150	C27H30O14	Exocarpium Citri Grandis
6	Naringin	442428	C27H32O14	Exocarpium Citri Grandis
7	Naringenin 7-O-glucoside	9910767	C21H22O10	Exocarpium Citri Grandis
8	Naringenin	932	C15H12O5	Exocarpium Citri Grandis
9	Azelaic acid	2266	C9H16O4	Panax ginseng
10	Ginsenoside Re	441921	C48H82O18	Panax ginseng
11	Ginsenoside Rf	441922	C42H72O14	Panax ginseng
12	Benzoylaconine	20055771	C32H45NO10	Aconitum carmichaeli Debx
13	Benzoylmesaconine	24832659	C31H43NO10	Aconitum carmichaeli Debx
14	Ginsenoside Rb1	9898279	C54H92O23	Panax ginseng
15	Ginsenoside Rg2	21599924	C42H72O13	Panax ginseng
16	Ginsenoside F2	9918692	C42H72O13	Panax ginseng
17	Acacetin	5280442	C16H12O5	Panax ginseng
18	Ginsenoside Rc	12855889	C53H90O22	Panax ginseng
19	Oxypeucedanin	160544	C16H14O5	Exocarpium Citri Grandis
20	Aurapten	1550607	C19H22O3	Exocarpium Citri Grandis
21	Tuberonic acid	6443968	C12H18O4	Panax ginseng

**Table 2:** Degrees of the top 20 targets.

Gene (target) name	Gene symbol	Degree
Tumor suppressor p53/oncoprotein Mdm2	TP53	121
Serine/threonine-protein kinase AKT	AKT1	114
Axin1/beta-catenin	CTNNB1	106
Tyrosine-protein kinase SRC	SRC	102
Heat shock protein HSP 90-alpha	HSP90AA1	101
Epidermal growth factor receptor erbB1	EGFR	99
Insulin-like growth factor I receptor	INS	97
MAP kinase ERK1	MAPK3	91
Signal transducer and activator of transcription 3	STAT3	90
Caspase-3	CASP3	87
Tumor necrosis factor-alpha	TNF	84
Vascular endothelial growth factor A	VEGFA	82
Mitogen-activated protein kinase 1	MAPK1	78
Interleukin-1 beta	IL1B	75
Cyclin D	CCND1	75
Hypoxia-inducible factor 1-alpha	HIF1A	70
PI3-kinase p110-alpha subunit	PIK3CA	67
PI3-kinase p85-alpha subunit	PIK3R1	63
Estrogen receptor alpha	ESR1	63
Peroxisome proliferator-activated receptor gamma	PPARG	61

RETRACTED

**Table 3:** Docking score between key targets and corresponding constituents.

Target	Gene symbol	Constituents	Docking score
Hypoxia-inducible factor 1-alpha	HIF1A	Apigenin	-5.96
Serine/threonine-protein kinase AKT	AKT1	Apigenin	-5.765
Serine/threonine-protein kinase AKT	AKT1	Naringenin	-4.455
MAP kinase ERK1	MAPK	Naringenin	-6.749
MAP kinase ERK1	MAPK	Tuberonic acid	-4.315
Glycogen synthase kinase-3 beta	GSK3B	Acacetin	-6.788
Glycogen synthase kinase-3 beta	GSK3B	Aurapten	-6.991
Glycogen synthase kinase-3 beta	GSK3B	Apigenin	-6.327
Glycogen synthase kinase-3 beta	GSK3B	Naringenin	-6.749
Glycogen synthase kinase-3 beta	GSK3B	Oxypeucedanin	-6.06
Solute carrier family 2, facilitated glucose transporter member 4	SLC2A4	Apigenin	-7.912

## Data Availability

The data that support the findings of this study are available from the corresponding authors upon reasonable request.
